# Acceleration of Deep Neural Network Training Using Field Programmable Gate Arrays

**DOI:** 10.1155/2022/8387364

**Published:** 2022-10-17

**Authors:** Guta Tesema Tufa, Fitsum Assamnew Andargie, Anchit Bijalwan

**Affiliations:** ^1^Faculty of Electrical and Computer Engineering, Arba Minch Institute of Technology, Arba Minch, Ethiopia; ^2^School of Electrical and Computer Engineering, Addis Ababa Institute of Technology, Ethiopia; ^3^School of Computing and Innovative Technologies, British University Vietnam, Hu'ng Yên, Vietnam

## Abstract

Convolutional neural network (CNN) training often necessitates a considerable amount of computational resources. In recent years, several studies have proposed for CNN inference and training accelerators in which the FPGAs have previously demonstrated good performance and energy efficiency. To speed up the processing, CNN requires additional computational resources such as memory bandwidth, a FPGA platform resource usage, time, power consumption, and large datasets for training. They are constrained by the requirement for improved hardware acceleration to support scalability beyond existing data and model sizes. This paper proposes a procedure for energy efficient CNN training in collaboration with an FPGA-based accelerator. We employed optimizations such as quantization, which is a common model compression technique, to speed up the CNN training process. Additionally, a gradient accumulation buffer is used to ensure maximum operating efficiency while maintaining gradient descent of the learning algorithm. To validate the design, we implemented the AlexNet and VGG-16 models on an FPGA board and laptop CPU along side GPU. It achieves 203.75 GOPS on Terasic DE1 SoC with the AlexNet model and 196.50 GOPS with the VGG-16 model on Terasic DE-SoC. Our result also exhibits that the FPGA accelerators are more energy efficient than other platforms.

## 1. Introduction

In recent years, deep learning has shown their usefulness and effectiveness in finding an answer to many actual world problems. The DNN, notably the convolutional neural network, is at the root of this renaissance. The convolution neural network was shown to be a useful tool for a variety of functions, including image classification [1], image recognition [2], and object detection [3]. A CNN involves a massive number of computations that it could profit from acceleration using GPUs and FPGAs [4, 5]. Deep CNN hardware implementations are constrained by a memory bottleneck that need numerous convolutions and fully connected layers, which necessitate a considerable amount of communication for parallel processing [6].

A variety of accelerators, including graphics processing units (GPUs), Field Programmable Gate Arrays, and application specific integrated circuits, has been used to increase the efficiency of CNNs [7–9]. Among these accelerators, GPUs are the most commonly employed to enhance throughput and memory bandwidth [8], both in the training and the inference process of CNN; however, they use high power [1, 6, 10]. An alternatively, field programmable gate arrays (FPGAs) are a natural option for neural network deployment since computing, logic, and memory resources may be merged into a single device. Based on FPGAs (field programmable gate arrays), CNN accelerators provide significant benefits because of their reduced power consumption, high throughput, and design flexibility [11]. FPGAs also provide high parallelism and exploit the features of neural network processing [12]. However, CNN on FPGA has a number of challenges such as requirements of memory storage, external memory bandwidth, and computational resource limitations. However, the FPGA restricted resources, such as the Stratix A7, have close effects to the midrange FPGA (Arria GX 10) citeli2017acceleration. The previous hardware accelerators for CNN have used different kernel for convolution and fully connected layers, which affect the FPGAs resource utilization [5, 13].

Intel's programmable solutions division has created a scalable convolutional neural network reference architecture for deep learning systems based on the OpenCL programming language. The OpenCL-based design tool is used to effectively accomplish the required accelerator design. This allows us to reuse the current code for Graphics Processing Units (GPUs) in FPGAs using OpenCL-based high-level synthesis tools [6, 14]. Developers may program the FPGAs in high-level languages like as C/*C*++ using high-level synthesis (HLS), which speeds up the development process. HLS techniques provide a developer with an extremely simple programming model as FPGA [12]. However, the CNNs are mostly solved using methods based on matrix-multiplication; this somehow requires the movement of huge volumes of data between compute units and external memory [5]. To speed up processing, the CNN requires more computational resources. Nonetheless, when processing CNNs, a memory bandwidth is often the bottleneck. Because of the high memory requirements of the fully connected (FC) layers, layer sections and the execution might be memory limited. The enormous number of weights held by these layers accounts for the high number of memory reads. If any of these accesses are to external memory, for instance, dynamic random access memory, throughput and energy power usage would be significantly impacted because dynamic random access memory accesses have far more latency and energy consumption than the compute itself.

However, memory storage, external memory bandwidth, and computing resource limits provide a number of challenges for CNN on FPGA.

The contributions of this work are as follows:

1. It proposes single kernel for both convolutional and FC layers, which improve memory bandwidth and hardware resource utilization.
2. Loop parallelization and single instruction multiple data (SIMD) have been applied.
3. To get maximum throughput, we use design space exploration method that leverages resource usage and throughput and is able to find the optimal architecture configuration, for CNN on FPGA.

## 2. Background

This section explains the basic theoretical basis for solving image classification problems. As such, we explain how hardware accelerators are used for image classification by first giving brief description of the hardware platforms and convolution neural network.

### 2.1. FPGA Architecture

FPGAs (Field Programmable Gate Arrays) were first used nearly two and a half decades ago. FPGAs are semiconductor devices that are built around a grid of configurable logic blocks (CLBs) interlinked via programmable interconnects. The FPGAs are programmable devices that offer a versatile platform for developing unique hardware capabilities at a reduced development cost [15]. The modern FPGA has two main parts: programmable logic blocks (ALMs) and logic components [12].  Figure 1 shows that the FPGA has a different configurable logic block (CLB) as well as input and output ports. The configurable logic block (CLB) is the basic repeating logic resource on an FPGA, which contains smaller components, such as flip-flops, look-up tables (LUTs), and multiplexers. The FPGA resources that allow connecting the FPGA target to other devices are the input and output (I/O). Input and output are to change analog or digital signals to or from a digital value so that we can process the signals using an FPGA target. The FPGAs logic capacity has been greatly increased because of advancements in process technology, making them a feasible implementation option for bigger and more sophisticated designs. Generally, the FPGA nature of logic and resource usage affects the FPGA device's space, speed, and power efficiency [16].

### 2.2. Intel FPGA SDK for OpenCL

A high-level abstraction for FPGA programming is provided by the Intel OpenCL SDK as one of the HLS tools. A concurrent program is built to von Neumann fixed structure as shown in a series of instructions for hardware acceleration that each computation generally requires the retrieval of instructions as well as the moving of data between register data and also the memory [17]. The Intel OpenCL SDK solution, on the other hand, provides a highly effective solution. Inside this model, the platform resources are customized to the algorithm being run [17].

Global memory is arranged as external memory in the FPGA device for the memory system in the Intel OpenCL SDK, which could be DDR3 synchronous dynamic random access memory as well as other memory [18].

### 2.3. Convolutional Neural Networks

CNN is a type of deep neural network that is very useful for classification. It takes an input and predicts a class tag for it. CNN typically consists of many layers, such as convolutional layers, ReLU layers, pooling layers, normalization layers, and fully connected layers. So, every layer will have its own input and output, with the input mapped to either a linear or nonlinear transformation of the output. Below are listed a descriptions of the individual layers.

#### 2.3.1. Convolutional Layer

The convolution layer parameters are made up of a series of learnable filters. Each filter has a small spatial footprint, but extending to the maximum depth of the input volume. CNN's most important layer is the convolutional layer. It is being used to retrieve the characteristics of the input image or the upper layer's feature map data [19]. The procedure is a three-dimensional convolution calculation based on input data and a huge variety convolution kernels, as well as the convolution operation is essentially a three dimensional multiply accumulate operation that could be described mathematically.

(1) $$\begin{array}{c} y_{out}\left(f_{o},y,x\right)=\overset{i-1}{\underset{i_{y}=0}{\sum }}\overset{i-1}{\underset{i_{x}=0}{\sum }}w_{l}\left(f_{o},i_{y},i_{x}\right)\times y_{i}\left(f_{i},y+i_{y},x+i_{x}\right)+b_{i}\text{,} \end{array}$$

in which *y*_*i*_(*f*_*i*_, *y*, *x*) as well as *y*_out_(*f*_*o*_, *y*, *x*) refers neurons as input extracted feature *f*_*i*_ but also extracted feature *f*_*o*_, respectively. *W*_*l*_(*f*_*o*_, *f*_*i*_, *y*, *x*) demonstrates the weights in the *l*^th^ layer which is combined with *f*_*i*_, as well as *b*_*i*_ would be a bias. The convolution filters are *i* × *i* in length.

#### 2.3.2. Rectified Linear Unit Layer

A recently proposed activation function in CNN is the Rectified Linear Unit (ReLU) that can be applied by thresholding a matrix at zero which is known to converge faster in training and has smaller computational complexity while the Sigmoid or tanh(x) activation functions involve expensive arithmetic operations [19]. The ReLU has become very popular in the last few years in convolutional neural network architecture. The equation of ReLU is very simple as follows:

(2) $$\begin{array}{c} f\left(x\right)=\max\;\left(0,x\right)\text{.} \end{array}$$

#### 2.3.3. Pooling Layer

As shown in Figure 2, the pooling layer is known as the down sample layer; it reduces extracted feature redundancy as well a network computational cost by minimizing extracted feature dimensions but rather effectively prevents overfitting. Pooling is among the common operators inside a convolutional neural network. Convolved extracted features are compressed in a pooling layer by a dataset obtained near the area feature values [20]. Because images have the regional property, this operation is possible. The spatial size of feature values is reduced after the pooling operation, resulting in fewer computational tasks to perform in the flowing layer. The pooling operator's most common options include max pooling as well as average pooling. The term “max pooling” refers to the following:

(3) $$\begin{array}{c} O\left(i,j\right)=\max\;\left[O\left(i_{o},j_{o}\right):i\underline{<}i_{o}<i+p,j\underline{<}j_{o}<j+p\right], \end{array}$$

in which *p* is the operator's length and (*i, j*) is the vertical and horizontal index.

#### 2.3.4. Fully Connected Layer

The fully connected layer is the classical component of a feed-forward neural network, wherein every element inside the max pooling is linked to every component in the output nodes. The extracted features of the convolutional as well as max pooling require the input image's distributed high-level attributes. The FC layers were designed to combine such extracted features in order to categorize the input into several classes. The forward throw of the *lth* FC layer is calculated as follows:

(4) $$\begin{array}{c} O^{l+1}=f\left(b^{l}+f^{l}+w^{l}\right)\text{,} \end{array}$$

where *O*^*l*+1^ is the output at *l*+1 layers, *f* is the activation function, *b*^*l*^ is the bias for *l*^*th*^ layers, *f*^*l*^ is the feature map in *l* th layers, and *W*^*l*^ is the weights at the *l*^*th*^ layers.

By adjusting the filter size of the convolution controller, an FC layer could be easily translated to the convolutional layer, which would be especially useful in practice.

#### 2.3.5. Backpropagation

Back propagation has performed two updates that are for the weights and the deltas [21]. We are looking to compute *∂E*/*∂w*_*m*,*n*_^*l*^ which can be translated as the measurement of how a single pixel alters *w*_*m*,*n*_ in the weight affects the loss function *E*. During forward propagation, the convolution operation ensures that the pixel *w*_*m*,*n*_ in the weight, between an element of the weight and the input feature map element that it overlaps; a contribution is made in all the products [20]. Convolution between the input feature map of dimension *H* × *W* and the weight of dimension *k*_1_ × *k*_2_ produces an output feature map of size (*H* − *k*_1_ + 1) by (*W* − *k*_2_ + 1). By applying the chain rule in the following way, the gradient component for the individual weights can be obtained [9].

(5) $$\begin{array}{c} \frac{\partial E}{\partial w_{m,n}^{l}}=\overset{H-k_{1}}{\underset{i=0}{\sum }}\overset{W-k_{2}}{\underset{j=0}{\sum }}\delta_{i,j}^{l}\frac{\partial x_{i,j}^{l}}{\partial w_{m,n}^{l}}\text{.} \end{array}$$

The summations represents a collection of all the gradients *∂*_*i*,*j*_^*l*^ coming from all the outputs in layer *l*.

## 3. Literature Review

Recent FPGAs had also provided a significant design space for a convolutional neural network due to an increase throughout FPGA fabric density as well as reducing transistor scale. The work by Tapiador et al. [6] implemented a depth-wise separable convolution with a high rate of resources and also significantly increases bandwidth as well as accomplishes a complete pipeline through parameter tuning and through a streaming data interface and the on ping-pong. In the work by Kaiyoua et al. [22], CNN models and CNN-based implementations have been distinguished. The requirements for memory, computation, and system reliability for mapping CNN on embedded FPGAs were summarized. Requirement analysis: they proposed Angel-Eye, which is a programmable as well as configurable CNN hardware accelerator combined with quantization method, compilation tool, as well as a data quantization technique. The compilation tool converts a specific CNN model into the hardware configuration. They were tested on the Zynq XC7Z045 platform and outperformed; peer FPGAs on same network have same of performance as well as power efficiency by6*x*and5*x*, respectively. In the work by Naveen Suda et al. [5], FPGA throughput is optimized on large-scale CNN with 3D convolution as matrix-multiplication. Their work demonstrated that ImageNet classification on the P395-D8 board can achieve a peak performance of 136.5 GOPS for convolution operations and 117.8 GOPS for the entire VGG network.

In terms of the processing time, the FPGA implementation has almost the same performance as the GPU implementations although the FPGA's memory bandwidth is much smaller and has much high energy efficiency than the GPU's one. FPGAs will be advantageous in the high-performance computing scope for these reasons because they provide reprogrammable hardware as well as low power consumption, and FPGA implementation is a cost effective also fast [12] while OpenCL enhances the code portable as well as programmable of FPGA, which greatly reduces the time and complexity programming process and it comes at the best of performance [8].

## 4. Methodology

In this section, we would go over the architecture in general, including convolution, input max pooling, and backward and output kernels.

### 4.1. Accelerator Design

The overall system design flow as well as both host and device system section of the OpenCL kernels is created with the Intel FPGA SDK for the OpenCL enhanced version channel. The hardware accelerators design has five kernels, such as forward convolution, backward convolution, pooling, input, and output. The input and output kernels have been used to transfer extracted features as well as weight from and to the main memory, which brings some kernels with high-throughput sequencing data. The convolution kernel is designed to speed up the most parallelize computations in CNNs, which typically include the convolution operation and the FC layer [7].

The Max-pool part works to dwindle the dimension of the information by combining the outputs of neurons into a single within the another layer and undersampling operations specifically on the yield data stream of the convolutional part. The cascaded kernels shape a channel, which can operate the essential CNN operations without the requiremet of putting away interlayer information backmost to external memory. So, every convolution channel has a computing unit, and the kernel is made up of many computing units to do parallel convolution [9]. Both of input and output kernels are a most vital kernel which are utilized for a data movement and a kernel that is outlined to bring or store information from or to a main memory for the computing path. The input kernels begin with such a global work items in convolution configuration whereas the output kernel is operating in an NDRange unveiling with global work items. To enable concurrent work group processing, the work items have been organized up into multiple running in parallel work groups, also with a local work group length of (*i*, *i*). The convolution filters size is 3 × 3, which minimizes computational costs and weight sharing that to lower back-propagation weights. The number of pixels shifted over the input matrix is referred to as the stride, and we use the stride size as 2 × 2 to modify the amount of movement over the image.

### 4.2. Forward Convolution Kernel

The forward convolution kernel performs a convolution operation. The forward convolution kernel performs a convolution operation. At each position, the multiplication between each element of the kernel and the input feature map element is computed and the results are summed up to obtain the output at that current location. The convolution operation is essentially a three-dimensional multiply accumulate (MAC) operation, which can be defined as

(6) $$\begin{array}{c} y_{o}\left(fe_{o},y,x\right)=\overset{C_{l}}{\underset{fe_{i}=1}{\sum }}\overset{i-1}{\underset{i_{y}=0}{\sum }}\overset{i-1}{\underset{i_{x}=0}{\sum }}w_{l}\left(fe_{O},i_{y},i_{x}\right)\times y_{i}\left(fe_{i},y+i_{y},x+i_{x}\right)+b_{i}, \end{array}$$

in which *y*_*i*_(*fe*_*i*_, *y*, *x*) as well as *y*_*o*_(*fe*_*o*_, *y*, *x*) refers neurons as input extracted feature *f*_*i*_ but also extracted feature *fe*_*o*_, respectively. *W*_*l*_(*fe*_*o*_, *fe*_*i*_, *y*, *x*) demonstrates the weights in the *l*^*th*^ layer which is combined with *fe*_*i*_, as well as *b*_*i*_ would be a bias.

### 4.3. Input Kernel

The algorithm 1 shows that the input kernel is used for reading input extracted features and relates filters from memory, along with feeding weight into the local buffer and obtaining extracted features and caching them in the local buffer. Because an input extracted feature is recycled by numerous different filters, the input array is cached in local memory for access during data processing and to reduce the access of global memory.

1. Get global and local index of work item
2. Calculate location for input features and filters using index
3. Bring input features into the local memory
4. Bring filter into the local memory
5. #progma unroll
6. for each component i in both input feature and filter do
7. Load weight into weight buffer
8. Fetch the weight and bias by fetcher
9. end for.

### 4.4. Pooling Kernel

The Pooling part performs to reduce the dimension of the weight by combining the outputs of neurons into a single within the another layer and undersampling operations specifically on the output data stream of the convolution kernel. The pooling layer reduces the convolutional outcomes while using the average or maximum value of elements in an area that is dependent on subsequent iterations. A shift registers with the depth that is developed for caching the accumulating data, similar to such convolutional layer. Then, depending on the pooling method, accumulating operations are performed on the shift register.

### 4.5. Output Kernel

The output kernel reads backproagation results from the accumulation channel and writes them back to global memory and then outputs to a local buffer, then extracts the data from the buffer, and copies it back to DDR. This work makes use of batch processing to reduce the time it takes for filters to be reused in FC layers. As a result, in the FC layer output kernel, N batch sets of results must be collected and written. It processes one set of results for the additional layer. The kernel is constructed in an NDRange manner, executing with work items in parallel, so the output processing is entirely independent.

### 4.6. Backward Convolution Kernel

This kernel reads the result from the max pooling buffer channel as well as performs two functions: error *δ* calculation and partial derivatives Δ W and Δ*E* calculation, both of which are cross-correlation processes. The cross-correlation operation can be implemented by reversing the data in the convolution kernel. The difference in resource usage is that while calculating the derivatives, we require two input buffers for both *δ*^*l*^ and *δ*^*l*−1^. Convolution between the input feature map of dimension *H* × *W* and the weight of dimension *k*_1_ × *k*_2_ produces an output feature map of size (*H* − *k*_1_+1) by (*W* − *k*_2_+1). By applying the chain rule in the following way, the gradient component for the individual weights can be obtained [9].

(7) $$\begin{array}{c} \frac{\partial E}{\partial w_{m,n}^{l}}=\overset{H-k_{1}}{\underset{i=0}{\sum }}\overset{W-k_{2}}{\underset{j=0}{\sum }}\delta_{i,j}^{l}\frac{\partial x_{i,j}^{l}}{\partial w_{m,n}^{l}}\text{.} \end{array}$$

## 5. Optimizations for Performance

In this section, we will discuss performance optimization techniques such as throughput maximizing, quantization, memory communication, parallelism in convolution neural networks, and converting fully connected layer to convolution layer.

### 5.1. Throughput

To keep moving forward, the accelerator's throughput, SIMD, and concurrent computing units are announced. The input kernel retrieves the SIMD and sends it to numerous computing units in the convolution. By adjusting the value of the SIMD as well as the number of computing units that is deployed, design could obtain scalable performance and hardware costs without requiring changes to the kernel code.

#### 5.1.1. Computing Unit

  The FPGA chip's resources are limited. If hardware resources are required for the optimization techniques, each kernel could have multiple compute units generated. This necessitates the creation of multiple copies of the various transmission lines. Even so, multiple computing units could not always improve throughput linearly since all computing units communicate over the global memory bandwidth. This causes memory access contention among computing units.

#### 5.1.2. Single Instruction Multiple Data (SIMD)

  To increase the data processing performance of an OpenCL kernel by processing various work items can be accessed by a single instruction multiple data (SIMD) approach without annually vectorizing the kernel code. The largest amount of work items per workgroup that the Intel FPGA SDK for OpenCL compiler could execute SIMD or vectorized was determined. The work group size that could be used is defined by the compiler, and the local work size argument is used to clEnqueueNDRangeKernel. The workgroup length can be allowed to pass to clEnqueueNDRangeKernel as such local work length argument. The above enables the compiler to adequately enhance the generated kernel code.

#### 5.1.3. Loop Unrolling

  The several loop iterations in the device code could have an impact on the kernel performance. The loop unrolling method could assign the most hardware resources and minimize or even eliminate the loop queue, that is, increase the throughput in a linear manner. This approach supports memory coalescing as well that also reduces memory transaction cost.

### 5.2. Quantization Technique

In general, artificial neural deployments, including convolutional neural networks, make use of a 32-bit floating point. The circumstance, even so, has been transformed. Several more latest FPGA works on convolutional neural networks had also centered to use the fixed-point representation of the extremely narrow bit width, which now has accuracy reduction [23–25]. However, nevertheless, low-bit reduction-based designs demonstrate exceptional performance and energy efficiency; this indicates that extremely low-bit width is an useful solution for higher efficiency design [23, 26, 27].

[IL.FL], from which IL seems to be the total number of integer bits and FL has been the total number of fractional bits would be a fixed-point number structure. The overall number of bits is calculated as the sum of IL and FL as well as the fixed-point number has an exactness of 2^−*FL*^ and the scope could be described this way: [−2^*IL*−1^ and 2^*IL*−1^ − 2^−*FL*^] [23]. The fixed point is the hardware-friendly as well as enables so much logic resources on FPGAs, allowing for increased parallel computing [28]. This even decreases the chip's memory usage and bandwidth needs. Even so, as in fixed-point deployment, we would use a fixed-point which was with static configuration to create cost effective and much more precise hardware kernels [15]. In overall, quantization is the most significant element in accelerating huge CNNs on the FPGA platform.

### 5.3. Memory Communication

Because several developments are limited by memory bandwidth, the other option is to use efficient memory access to reduce communication cost. Several developments are limited by memory bandwidth, the other option is to use efficient memory access to reduce communication costs.

#### 5.3.1. Memory Alignment

  Here, on host side, memory allocated would have to be at least 64-byte aligned. This significantly improves the transmission efficiency of DMA transmitting on the host-FPGA communication. The allocation can be executed in Linux using the POSIX mem-align function, which is supported by GCC, or Windows use that aligned malloc function, which is held by Microsoft.

#### 5.3.2. The Local Memory Caching

  Global memory, constant memory, local memory, and private memory are the four areas of the OpenCL memory model. Local memory, which would be executed in the on-chip Random access memory block, does have significantly decreased latency and high bandwidth than main memory. As a result, we can cache global memory which requires multiple accesses previous to computation using local memory. Those certain cached local memories have been viewable to everyone, work items in the same workgroup when data parallelism is enabled. By minimizing the memory access, the use of local memory would improve kernel performance.

### 5.4. Parallelism in Convolutional Neural Network

Those processing, which would include reading, convolving, pooling, and writing back, are data independent of varying extracted features. As a result, the entire output extracted feature can be vectorized along the N dimension, with each section processed on a different data path. This can be executed by a computing unit in OpenCL that would significantly enhance the proposed design throughput [10]. Furthermore, every convolution operation of an extracted feature unit consists of stage element-wise multiplication of input extracted feature and filters, followed by the accumulation of the product of these operations. [19]. In the first process, multiplication is completely independent and could be performed using a data parallelism technique.

### 5.5. Changing FC Layers to Convolution Layers

Fully connected layers and convolution layers have the same working order form, which entailed multiplying and adding. It should be noted that because the only difference between the fully connected and the convolution layer would be that the neurons in the convolution layer are only connected to a local region at the input and that many of the neurons in the convolution layer volume share parameters. The fully connected (FC) layer operates on a flattened input, with each input connected to all neurons. Dot products, on the other hand, are always computed by neurons in both layers, so their functional form is similar. There are two approaches for changing FC layers to convolution layers. First, choose a convolution layer kernel filter with the same length also as input feature's map, and secondly, by using 1 × 1 convolutions with multiple channels.

## 6. Experimental Setup

The Terasic DE1 SoC Development Kit (DK) of FPGA board is used to implement the experiments. DE1 SoC would be a powerful hardware design platform based on Intel System-On-Chip (SoC) FPGA. The DE1 SoC board uses several features which enable designer to complete a broad range of designing circuits projects.

The terasic DE1 SoC board has M10K-10-kbit memory blocks including soft error correction code (ECC), as well as a 400 MHz/800 Mbps interface of an external memory and 64 MB of the SDRAM, 1 GB (2 × 256M × 16) of DDR3, and micro SD card port on Hard Processor System (HPS) memory [29]. The Intel cyclone V SoC 5CSEMA5F31C6 has 85K programmable logic elements, 4,450 Kbits of memory embedded, 6 fractional phase locked loops (PLLs), dual-core ARM Cortex-A9 (HPS), and 2 memory controllers based on TSMC's 28-nm low power (28LP) process technology. The architecture of a DE1 SoC includes two USB 2.0 Host ports (ULPI interface with USB type A connector) [29]. As communication ports, connectors, displays, switches, buttons, indicators, audio, and video inputs, G-Sensor on HPS and UART to USB (USB Mini-B connector), 10/100/1000 Ethernet, PS/2 mouse/keyboard, IR emitter/receiver, and I2C multiplexer are used. The accelerator boards communicate with the host through the use of an 8-lane PCI express link.

We use Intel SDK for OpenCL intelFPGA_Standard_18.1.0 build 625. The Intel FPGA SDK for OpenCL Standard Version includes programs, drivers, development kit library resources as well as files, and much more. The Intel SDK for OpenCL Standard_18.1.0 has logic components such as offline Compiler translates, a set of commands, host runtime providing the OpenCL host, and runtime API for the OpenCL host code. We used the Board Support Package (BSP) 18.1 version for de1soc board BSP from Terasic and Intel SDK for OpenCL the intelFPGA_Standard_18.1.0 with 625 buildings is used. Additionally, (Intel® CoreTM i5-4300) CPU and (AMD Radeon (TM) R5 M330) GPU are used.

## 7. Result and Discussion

In this section, we evaluate the performance of our proposed system with the different design specifications. The objective of this exercise is to learn the resource utilization and performance figures for combinations of design specifications. We employ two well-known CNN models for the possible combinations of convolutional neural network design specifications.

### 7.1. Design Performance and Analysis

We advanced to evaluate the accuracy of our design on the ImageNet ILSVRC-2012 data set, where it contains up to 1.2 million training and 50k validation instances. An AlexNet Caffe model, that has 61 million parameters as well as a top-1 accuracy of 57.2% and a maximum classification of top-5 accuracy of 80.3%, has been used as a reference model. On the same ILSVRC-2012 data set, we furthermore examined a larger, more latest network, VGG-16 [30]. The VGG-16 does have 138 million parameters and much more convolutional layers, but still only three fully connected layers at the moment [12]. The accuracy of our work was assessed with executing our models on 728K training and 50K validation samples from the ImageNet 2012 data set. The accuracy comparision for AlexNet model in Figure 3 and the accuracy comparision for VGG-16 model demonstrate the accuracy of various quantization compression rates.

Figure 3 and Figure 4 demonstrate the accuracy of various quantization compression rates. As shown, the model's accuracy starts to decline considerably while compressing below 8-bit data quantization of its base accuracy. The difference between the Caffe tool using AlexNet model with 32 bit floating point and the 32 bit floating point FPGA design on top-1 and top-5 accuracies is 0.5% and 0.59%, respectively. The difference between a 16-bit fixed point Caffe tool and FPGA design on top-1 accuracy is 0.59% and top-5 accuracy is 0.9% accuracy loss compared to the reference design. The accuracy difference between 8 bit Caffe and FPGGA implementation design on top-1 and top-5 accuracies is 0.77% and 0.5%, respectively. The accuracy difference between 4 bit Caffe tool and FPGGA implementation design on top-1 and top-5 accuracies is 2.05% and 1.19%, respectively. Therefore, the accuracy of our implementation is excellent. As a result, the exactness of our implementation is comparable to baseline.

### 7.2. Computation Throughput and Energy Efficiency

In this subsection, we will discuss the computation throughput as well as the energy efficiency of the system. Figures 5 and 6 show throughput, and Figures 7 and 8 depict energy efficiency.

### 7.3. Computation Throughput

In Figures 5 and 6, our experiments have show that with low-bit width quantization, we can achieve a high throughput in results. The low-bit width quantization techniques have significant benefits because it allows for high memory cache to be used as well as removes memory constraints in deep learning methods. This enables faster data movements and more efficient computation of the throughput in hardware acceleration. And it enables the device to do more operations per second, significantly speeding up workloads. Because of these advantages, low-bit width implementations are likely to become common in training and inference, particularly for convolutional neural networks.

### 7.4. Computation Efficiency

Figures 7 and 8 demonstrate that the low-bit width quantizataion neural networks improve power efficiency. As we have discussed in the subsection of computation throughput, it reduces memory access costs by enabling high memory cache usage and increasing compute efficiency. Using low-bit quantization can reduce power consumption and save significant energy. Low-bit width quantization uses less energy and enhances compute efficiency, resulting in lower power consumption. Furthermore, decreasing the number of bits used to represent the neural network's parameters results in less memory storage.

Generally, among all the data quantization as observed from Figures 5 to 8, low-bit width-based designs demonstrate exceptionally good speed and energy efficiency. This indicates which extremely low-bit width is a likely answer for high performance. However, the extremely low-bit width has accuracy reduction.

### 7.5. Resource Utilization

Table 1 shows the trained CNN on FPGA resource usage. During training, CNN on FPGA consumes huge computational resources. We trained our models on the de1_SoC board before changing any parameters, and the resource usage is illustrated in Table 1.

Our design, as stated in section III, includes two major variables: the number of computing units and the number of SIMD. The replication of full data paths is the total number of computing units, that also controls the balance among both resource usage. Additionally, a compute unit may be composed one or more processing elements depending on our design choice. Having more processing elements per compute unit can significantly raise the data processing speed by allowing single instruction multiple data (SIMD) execution mode.

The number of SIMD processing elements is a design choice that also allows for contiguous memory retrieval which can enhance memory utilization efficiency. In the design, we were using a static configuration number of SIMD units, which allowed us to work with restricted on-board resources. We investigate how well the number of computing units and SIMD impact the De1 Soc-based board's resource utilization and throughput.

In order to achieve the maximum performance of our design, we configured the SMID as fixed as well as varied the number of computing units. When both parameters grow, there is also a growth in resource usage. Furthermore, with data path replication in the framework, the number of computing units does have a greater effect on resource utilization than that of the number of units. Whenever these variables are increased, it is simple to see even a linear improved performance in throughput. However, because of the limited resources on the DE1 SoC, the integration of computing is equal to sixteen as well as SMID sixteen results in successful synthesis both on fixed point and floating point.

### 7.6. Power Measurement

The power consumption is an important element in hardware accelerator performance. The power drain on one of the devices tells us how hard it is working and how power-intensive the design would be. This is especially essential for evaluating deep learning applications for hardware accelerators, where power consumption is a major consideration. We measure performance and power consumption by using the Perf performance analysis tool for Linux. The idle CPU-only system absorbs 50.70 W before the FPGA accelerator board is installed on the system. When using Caffe tools to run AlexNet and VGG-16 models, the average power utilization starts to rise to 109.2 W. Whenever a DE1 SoC-based FPGA board is properly configured, the idle power consumption rises to 63.40 W. Throughout CNN kernel implementation, the overall power usage of the hardware acceleration rises to 78.2 W by averages. Thereby, a power use for running a CNN framework on the a DE1 SoC-based board is (78.20–50.70) = 27.5 W.

### 7.7. Comparative Discussion on Previous Work and Other HPC Platform Design

In this section, we would first compare our implementations with previous FPGA research. The following is a comparison with similar designs focused on other high-performance computing platforms, such as CPUs and also GPUs.

#### 7.7.1. FPGA-Based Design

We contrast the proposed models' efficiency to that of a number of other recent FPGA-based CNN design features. To determine the throughput, divide the total floating point numbers or fixed-point operations through the entire execution time and then use GOP/S as a unit for floating point as well as fixed-point operations in our implementation design. Zhang et al. [31] implemented a convolution layer which obtained 61.62 GOPS again for single precision floating point design. Similarly, the work by Yufei Ma et al. [13] reported 134.1 GOPS and 117.3 GOPS on a convolution layer for AlexNet and NIN model, respectively, while they achieved the overall performance 114.5 GOPS and 117.1 GOPS for AlexNet and NiN model, respectively. Our throughput from the 4-bit fixed point on DE1_SoC for AlexNet model 203.75 GOPS and also for VGG-16 model 196.50 GOPS on DE1_SoC. Our work gained 1.78x more throughput over the work by Naveen Suda et al. [5] with only using 85 DSP blocks. Furthermore, our design outperforms the RTL design in [13] by 1.51x on the different boards, demonstrating that OpenCL-based designs can compete with RTL designs. When compared to other designs, our DE1 SoC design has had the highest throughput, and there is still room for improvement.

#### 7.7.2. Other HPC Platform-Based Design

We as well introduce energy consumption as both a measure for evaluation, which would be the ratio of throughput to power consumption (GOPS/Watt). In terms of throughput, the GPU is the best alternative, followed by one FPGA design, as shown in Table 2. Power usage, on the other hand, is an important measure to take into account in modern digital design. The GPU absorbs 3.709X so much energy than that of the FPGA, and the FPGA is 22.613x more efficient than the CPU.

## 8. Conclusion

In this work, we show a training and classification of a deep neural network that use the Intel, FPGA OpenCL SDK. To determine the best design requirements to speed up the CNN model for training while using constrained FPGA resources, we proposed a design space exploration methodology for energy efficiencies and resource utilization. We implemented CNN models such as AlexNet and VGG on the DE1 SoC FPGA board using the proposed approach as well as gained higher performance when compared to earlier work. As we compared with the other platform, the CNN training on FPGA consumes less power consumption and training time. Our findings indicated that FPGAs could obtain greater power or energy efficiency than GPUs, which typically restrict improvement only to power efficiency. We noted that it is mainly due to the huge difference in maximum compute performance as well as the external memory bandwidth between FPGAs and GPUs.

Generally, our designs achieve 203.75 GOPS on Terasic DE1 SoC with the AlexNet model and 196.50 GOPS with the VGG-16 model on Terasic DE-SoC. This, as far as we know, outperforms existing FPGA-based accelerators. Compared to the CPU and GPU, our design is 22.613X and 3.709X more energy efficient, respectively.

## Figures and Tables

**Figure 1:** Overview of FPGA architecture, taken from [16].

**Figure 2:** Max pool, taken form [19].

**Figure 3:** The accuracy comparison for AlexNet model.

**Figure 4:** The accuracy comparison for VGG-16 model.

**Figure 5:** Throughout with difference data quantization with Caffe [CPU].

**Figure 6:** Throughput with difference data quantization on FPGA.

**Figure 7:** Energy efficiency with difference data quantization with Caffe [CPU].

**Figure 8:** Energy efficiency with difference data quantization on FPGA.

**Table 1:** Resource usage CNN training.

Data quantization (bit)	ALUTs	DSP	FFS	M10 K
32	139913	85	172677	497
16	108313	76	144798	422
8	88712	64	126918	346
4	74511	52	91158	187

**Table 2:** Compare with other devices.

Platform	CPU	GPU	FPGA
	Intel® Core i5-4300	AMD Radeon (TM) R5 M330	DE1_SoC
Technology	22 nm	28 nm	28 nm
Power (Watt)	58.5	94.50	18.5
Throughput (GOPS)	28.50	280.60	203.75
Energy efficiency (GOPS/W)	0.487	2.969	11.013

## Data Availability

The source of the author's framework along with the datasets and analysis during the current study is already publicly available on https://image-net.org/challenges/LSVRC/2012/index php which is maintained by Princeton University and Stanford University. Quartus-18.1.0.625 software was used for processing and classification purposes during the author's research experiment.
